# Unraveling the Nanoscopic Organization and Function of Central Mammalian Presynapses With Super-Resolution Microscopy

**DOI:** 10.3389/fnins.2020.578409

**Published:** 2021-01-08

**Authors:** Lia G. Carvalhais, Vera C. Martinho, Elisabete Ferreiro, Paulo S. Pinheiro

**Affiliations:** ^1^Center for Neuroscience and Cell Biology, University of Coimbra, Coimbra, Portugal; ^2^Center for Innovative Biomedicine and Biotechnology, University of Coimbra, Coimbra, Portugal; ^3^Institute for Interdisciplinary Research, University of Coimbra, Coimbra, Portugal

**Keywords:** super-resolution microscopy, presynaptic structure, active zone, vesicle exocytosis, neurotransmitter release

## Abstract

The complex, nanoscopic scale of neuronal function, taking place at dendritic spines, axon terminals, and other minuscule structures, cannot be adequately resolved using standard, diffraction-limited imaging techniques. The last couple of decades saw a rapid evolution of imaging methods that overcome the diffraction limit imposed by Abbe’s principle. These techniques, including structured illumination microscopy (SIM), stimulated emission depletion (STED), photo-activated localization microscopy (PALM), and stochastic optical reconstruction microscopy (STORM), among others, have revolutionized our understanding of synapse biology. By exploiting the stochastic nature of fluorophore light/dark states or non-linearities in the interaction of fluorophores with light, by using modified illumination strategies that limit the excitation area, these methods can achieve spatial resolutions down to just a few tens of nm or less. Here, we review how these advanced imaging techniques have contributed to unprecedented insight into the nanoscopic organization and function of mammalian neuronal presynapses, revealing new organizational principles or lending support to existing views, while raising many important new questions. We further discuss recent technical refinements and newly developed tools that will continue to expand our ability to delve deeper into how synaptic function is orchestrated at the nanoscopic level.

## Introduction

Imaging in neurosciences has come a long way since 19th-century neuroanatomist Ramon y Cajal made detailed drawings of silver-stained neurons and postulated that they were not continuous, but instead connected through gaps. These would be known as synapses. Synapses were first visualized in detail in the 1950s (e.g., Palay, 1956) and are believed to be the sites where learning and memory are molecularly encoded (Mayford et al., 2012). Classical optical microscopy techniques have been paramount for our understanding of the structural and molecular organization of neurons. However, the more we learn about their intricate features, the more the limitations of these techniques become apparent. While electron microscopy has provided exquisite structural details of membrane-limited or electron-dense synaptic structures, it cannot adequately resolve their crowded molecular composition or be used in live specimens and is technically demanding. Fluorescence microscopy, on the other hand, is a less demanding technique that can be used in live tissues and provides the ability to determine the abundance, cellular localization, interactions, and dynamics of specific molecules, by resorting to direct or antibody-mediated multi-color target labeling and simultaneous imaging (Lichtman and Conchello, 2005). However, as powerful as conventional fluorescence microscopy techniques have become, they are generally limited to a resolution of roughly half the excitation wavelength (a couple hundred nanometers) and are, therefore, unable to properly resolve the subcellular neuronal structures that most interest neurobiologists, notably synapses, subsynaptic compartments, and their underlying molecular complexes and nanodomains. Unraveling their detailed molecular composition and functional dynamics (for example, the trafficking of receptors or channels at the membrane or the changes in protein cluster number or size with synaptic activity) requires imaging at the nanoscale, using so-called super-resolution microscopy (SRM) techniques, that were developed to surpass the diffraction-limited resolution of conventional light microscopy while attempting to retain its versatility. Owing to the evolution of fluorophores and both hardware and software, many SRM techniques have been successfully and routinely used in biology for live-cell imaging (e.g., Godin et al., 2014) and applied to neurons.

Neurons are arguably the most compartmentalized cells in nature. At chemical synapses, neurotransmitters are released from presynaptic terminals in an extremely fast and precisely timed manner to activate neurotransmitter receptors on the postsynaptic neuron (Südhof, 2013). The entire process requires complex, spatially restricted, and often stoichiometrically defined interactions between specific sets of proteins (Patrizio and Specht, 2016) whose structural organization, dynamics, and expression levels are critical for the function of neuronal circuits (Emes and Grant, 2012). Electrophysiology techniques have been paramount to our understanding of synaptic function, since they provide unsurpassed temporal resolution for detecting the electrical changes produced by the activation of neurotransmitter receptors or ion channels, and have even allowed direct recordings from small presynaptic terminals (Novak et al., 2013). However, they don’t provide any spatial or dynamic information regarding the molecular players involved in synaptic activity and plasticity, creating the need for correlative structural data. This is where SRM techniques provide unique advantages for studying synaptic function over diffraction-limited microscopy or fixed-sample-only electron microscopy. In the following sections, we begin with a brief description of the most common SRM techniques. We then review how SRM has shed light on the molecular complexity and structural features of presynaptic neuronal compartments of central mammalian synapses, and how protein distribution, nanoclustering, and dynamics shape neuronal signaling. We finish by presenting recent developments in SRM that will, undoubtedly, continue to revolutionize synapse biology. We apologize in advance for any omissions that may have been made due to space constraints or to our focus on central mammalian synapses.

## Brief Overview of Super-Resolution Imaging Methods

Super-resolution fluorescence microscopy techniques can be broadly divided into two main categories: deterministic and stochastic. Deterministic SRM techniques are based on exploiting non-linear interactions of fluorophores with light, using patterned illumination, to limit the focal spot size. Among these techniques, we find structured illumination microscopy (SIM) and its variations, stimulated emission depletion (STED) and reversible saturable optical fluorescence transition (RESOLFT) microscopy. STED pioneered these techniques by combining an excitation laser beam with a second, donut-shaped, laser beam with a red-shifted emission wavelength (depletion or STED beam) with ideally zero intensity at the center ring. This second beam suppresses peripheral excitation by quenching excited fluorophores, thereby limiting fluorescence emission to its centermost part and allowing resolutions well below the diffraction limit (Klar and Hell, 1999; Klar et al., 2000). STED is versatile for imaging fast cellular events but can be costly to implement, and there is limited fluorophore choice due to the high laser intensities that are required. RESOLFT is based on a similar illumination principle but employing photoswitchable emitters (Hofmann et al., 2005), namely photostable reversibly photoswitchable fluorescent proteins. In SIM, the samples are illuminated with a grating pattern that shifts phase over several frames to produce a *moiré* pattern. The results of this pattern are processed and reconstructed into images with an approximately two-fold improvement in resolution (Gustafsson, 2000). SIM can be used with conventional dyes in multi-color imaging and yield high-speed acquisition frame rates for monitoring live cell dynamics (Kner et al., 2009; Lefman et al., 2011), but requires a dedicated microscope and substantial computation for image reconstruction. SIM is best suited to thin samples and the gain in resolution is smaller than with other techniques. However, non-linear SIM (NL-SIM), which uses a photoswitchable protein and low irradiation intensities, allows a resolution of 50 nm in biologically compatible imaging conditions (Rego et al., 2012). The higher resolutions achievable with STED and RESOLFT, which are based on laser scanning (as in confocal microscopy), come at the tradeoff of speed. However, parallelized acquisition strategies have allowed for much faster imaging rates (Chmyrov et al., 2013; Yang et al., 2014). STED also uses much higher laser intensities than RESOLFT (Hofmann et al., 2005; Willig et al., 2007), which can be a concern in long studies in living preparations and cause significant photobleaching and phototoxicity. To overcome these limitations, a new variation of 3D-STED, termed super-resolution shadow imaging (SUSHI), was recently developed (Tønnesen et al., 2018). SUSHI is based on imaging the extracellular space with diffusible dyes, thereby producing super-resolved negative images of all cellular structures that can reveal the micro-anatomy of living brain tissue, including dendritic spines and the synaptic cleft. This technique holds great promise for the future study of the dynamic processes associated with development and with synaptic activity and plasticity. It is also insensitive to photobleaching and poses less phototoxicity concerns due to the extracellular labeling, allowing for prolonged imaging sessions on large fields of view.

Stochastic methods, on the other hand, are based on the precise localization of the emitting fluorophores by temporally separating the activation of individual molecules in successive rounds of frame acquisitions (hence, they are also referred to as single-molecule localization methods). These methods include photoactivatable localization microscopy (PALM), stochastic optical reconstruction microscopy (STORM), and universal point accumulation for imaging in nanoscale topography (uPAINT) and can achieve resolutions well below the diffraction limit. PALM and STORM use a somewhat similar principle to achieve their high resolution but, whereas the first was developed using photoactivatable, genetically encoded fluorescent proteins fused to the protein of interest (Betzig et al., 2006; Hess et al., 2006), the later used pairs of organic fluorophores linked to antibodies (Rust et al., 2006). In PALM, specific illumination wavelengths are used to stochastically activate only a small subset of molecules, which are imaged and returned to a dark state, and the process repeated over many photoswitching iterations. In STORM, fluorophores are driven into a dark state in the absence of oxygen, from which a small number stochastically recovers and is imaged, and the process is also repeated over many iterations. Though these images are still diffraction-limited, mathematically localizing the center of the sparse fluorescent spots generates coordinates for each molecule, with a pointing accuracy of detection dependent on the square root of the intensity of the collected signal. Over-accumulation of all the detections is then used to obtain a pointillistic representation of all individual positions across all acquired frames (Betzig et al., 2006; Hess et al., 2006; Rust et al., 2006). This yields a merged image that contains the high-resolution information from the processed frames. One of the main advantages of PALM lies in the simplicity of its implementation, requiring basic molecular manipulations for expression of photoactivatable proteins fused to the targets of interest, simple imaging systems with suitable lasers, and analysis software that can be found for free. However, both PALM and STORM usually require very large numbers of iterations to reconstruct a single image, making them rather slow (minutes to tens of minutes per complete acquisition). Additionally, fluorophore photostability is a concern and the methods are prone to artifacts due to the complex post-acquisition processing for image reconstruction. Conceptually similar to STORM, direct STORM (*d*STORM) was developed using conventional cyanine dyes that can efficiently and reversibly photoswitch between dark and fluorescent states. This provides a simpler method that does not require the presence of activator fluorophores and does not rely on specific ratios and distances between two fluorophores attached to antibodies (Heilemann et al., 2008). Many organic fluorophores can be made to photoswitch in the presence of reducing buffers and are suitable to use in *d*STORM (Endesfelder and Heilemann, 2014). Finally, uPAINT, developed as a variation of PAINT (Sharonov and Hochstrasser, 2006), is based on imaging the real-time stochastic interaction of a specific fluorophore-coupled ligand with its target molecule (Sharonov and Hochstrasser, 2006; Giannone et al., 2010, 2013) by continuously and stochastically labeling while imaging. When such interaction occurs, the diffusion of the fluorophore is reduced, making it more likely to be detected than unbound fluorophores under specific illumination and imaging conditions. uPAINT allows following the trajectories of many single molecules simultaneously and for extended periods of time, but is limited to membrane-localized molecules. More recent variations employ fluorophore-labeled DNA oligos that bind to their unlabeled complementary sequences (DNA-PAINT; Jungmann et al., 2014). The different SRM methods have been thoroughly reviewed elsewhere (e.g., Godin et al., 2014; Sydor et al., 2015; Wu and Shroff, 2018; Dietz and Heilemann, 2019; Huszka and Gijs, 2019; Schermelleh et al., 2019) and a detailed breakdown of the features, advantages, and disadvantages of each has been published while this manuscript was under writing (Jacquemet et al., 2020).

## Super-Resolution Imaging of the Presynapse

Presynaptic active zones—the sites where neurotransmitters are released—are dynamic structures where molecular and functional changes are responsible for the regulation of neurotransmitter release and trigger several forms of short- and long-term synaptic plasticity (Choquet and Triller, 2013). Neurotransmitter release occurs with nanoscale and sub-millisecond precision and is orchestrated by the molecular interactions between a defined set of proteins forming the so-called SNARE complex, composed of Synaptosomal-Associated Protein, 25 KDa (SNAP25), synaptobrevin and syntaxin-1, and requires additional players such as Munc13, Munc18, complexins, and synaptotagmins acting as calcium sensors (Südhof, 2012). Exocytosis is then followed by the retrieval of proteins and membrane through endocytosis. At vertebrate central synapses, active zones are disk-like structures with a diameter of 200–500 nm; synaptic vesicles are only ∼40 nm in diameter and the protein complexes driving their fusion are smaller still. An elegant study, combining quantitative proteomics, STED microscopy at ∼40 nm resolution and 3D modeling, reconstructed the “average” presynaptic bouton as a structure of 0.37 μm^3^ containing approximately 380 vesicles and an astonishing 300,000 densely packed proteins that were modeled in atomic detail according to their known structures (with copy numbers ranging from a few tens to over 20,000), and distributed according to SRM imaging data (Figure 1) (Wilhelm et al., 2014). Even though only 60 proteins were included in the 3D model, this clearly illustrates how the precise localization, spatiotemporal interaction, and dynamics of active zone components remain far beyond the reach of conventional microscopy techniques in such a small and crowded environment. By complementing the detailed ultrastructural data provided by electron microscopy, studies resorting to SRM—though still relatively few—have contributed important insights into the molecular composition, organization, and dynamics of the presynaptic active zone.

**FIGURE 1:** Reconstruction of an average presynaptic terminal from purified synaptosomes. **(A)** Following a synaptosome purification procedure, serial electron micrographs were used to determine organelle numbers, sizes, and positions and reconstruct entire synapses. Shown is a single synaptosome representing the average physical parameters, with vesicles illustrated in dark beige, the active zone in red, larger organelles in dark gray, and mitochondria in purple **(B)** Section through the synaptic bouton showing the localization and abundance of 60 distinct proteins. Using information on protein copy numbers and their positions obtained by STED microscopy and other sources, they were placed in this synaptic structure in atomic detail. The reconstructed image reveals a densely crowded synaptic space, particularly around the active zone and vesicle cluster. Adapted, with permission from Wilhelm et al. (2014).

### Nanoarchitecture of Active Zones

At fast inhibitory and excitatory mammalian central synapses, several active zone scaffolding and tethering proteins have been identified, including Piccolo, Bassoon, Rab3-interacting molecule (RIM) and RIM-binding proteins (BPs), ELKS and Munc13, which are believed to connect vesicles to the plasma membrane and define the sites of exocytosis (Südhof, 2012). A first SRM study to look at the distribution of presynaptic proteins used multi-color 3D-STORM in mouse brain tissue sections to achieve a localization precision of 14 nm in the lateral plane and 35 nm in the axial plane (Dani et al., 2010). Both Piccolo and Bassoon, two active zone proteins that may have evolved to perform specific functions in vertebrate synapses, were found to have a similar axial distribution and to be organized in a highly oriented and extended manner, perpendicular to the active zone, with their C-termini pointing toward the presynaptic membrane and at distances close to 50 nm from it. Similar axial distributions were observed in subsequent studies using STED (Wong et al., 2018) or 3D-STORM (Trotter et al., 2019). The seemingly ubiquitous presence and precise arrangement of Bassoon at presynaptic active zones have made it a bona fide marker for the localization of other proteins with respect to active zones in many subsequent SRM studies. However, Bassoon itself may be implicated in synaptic modulation, since differences in its density in individual Bassoon clusters seem to explain the differences in the strength of presynaptic Cannabinoid receptor type 1 (CB1R) modulation between perisomatic and dendritic GABAergic terminals in the hippocampus (Dudok et al., 2015). Additionally, using dual-color dSTORM, Bassoon was shown to segregate from Ca_*v*_2.1 and RIM clusters and to suffer an activity-dependent unclustering at hippocampal synapses, with a concomitant increase in Bassoon nanodomains, which allow the recruitment of multiple active zone components (Glebov et al., 2017). This demonstrates that the macromolecular crowding of the active zone limits presynaptic function and that dynamic unclustering can be used to change presynaptic strength. A similar localization and organization of Bassoon at active zones was demonstrated using X10 expansion microscopy (Truckenbrodt et al., 2018), a technique that achieves its high resolution by physical sample expansion through embedding into swellable gels, instead of using advanced microscopy methods (see below).

In a more recent study using 3D-STORM, RIM1/2 was found to be more clustered than Munc13 or Bassoon and to preferentially localize at the center of synapses (Tang et al., 2016). RIM cluster numbers and size paralleled those of postsynaptic density protein 95 (PSD95) clusters, whereas Munc13 clusters were more abundant and widely distributed, and Bassoon clusters less abundant and more uniformly distributed. Using PALM, the distribution of RIM nanoclusters was found to closely match vesicle fusion sites and to align trans-synaptically with nanoclusters of PSD95 and glutamate receptors while extending even deeper into the postsynaptic structure (Tang et al., 2016). These results support the notion of a trans-synaptic nano-column aligning presynaptic regions of high vesicle fusion probability to postsynaptic regions of high receptor density at excitatory synapses. A subsequent study using multi-color STED at excitatory synapses, both *in vitro* and *in vivo*, showed a correlation between dendritic spine size and the number of aligned *trans*-synaptic modules, further supporting the notion of a precise trans-synaptic alignment. Though the number (but not the size) and dynamics of these modules changes rapidly with synaptic plasticity, they remain aligned (Hruska et al., 2018). These results also suggest that structural plasticity linked to synaptic potentiation could be mediated by addition of building blocks made of unitary synaptic nanomodules. It would be interesting to investigate if a reverse mechanism operates in synaptic depression. Using multi-color 3D-SIM, a similar trans-synaptic organization was also found at inhibitory synapses. Here, presynaptic RIM subsynaptic domains align opposite to postsynaptic γ-aminobutyric acid (GABA)_A_ receptor and gephyrin subsynaptic domains (Crosby et al., 2019). The number and volume of RIM clusters correlates with the number and volume of GABA_A_ receptor and gephyrin clusters at individual synapses, with a significant pairing between the pre- and postsynaptic structures, independently of synapse size. However, presynaptic structures positive for the vesicular GABA transporter do not show such correlation and are thus not representative of the active zone (Crosby et al., 2019). Therefore, similarly to glutamatergic synapses, GABA_A_ receptors and RIM at inhibitory synapses display a spatial segregation that strongly suggests a trans-synaptic coupling between them, likely reflecting the functional similarities between both synapse types, that is, optimized for fast ionotropic synaptic transmission. Identifying the molecular players involved in this *trans*-synaptic alignment will be important to better understand the coupling between pre- and postsynaptic function, and synaptic adhesion molecules, such as neurexins and neuroligins, are likely candidates. Indeed, using 3D-STORM, the adhesion molecule neurexin-1 was found to concentrate at presynaptic membranes within the synaptic cleft and to form discrete nanoclusters at a subset of excitatory synapses in both cultured neurons and hippocampal sections, which increased in size with development (Trotter et al., 2019). Typically, however, only one neurexin-1 cluster is found per synapse and only at a subset of synapses, which is incompatible with the widespread presence of trans-synaptic nanocolumns proposed to align sites of presynaptic vesicle fusion to postsynaptic receptor nanoclusters (Tang et al., 2016). Notwithstanding, expression of a C-terminal truncated neuroligin-1—the postsynaptic partner of neurexin—in neurons delocalizes it from α-amino-3-hydroxy-5-methyl-4-isoxazolepropionic acid (AMPA) receptor nanodomains and perturbs the trans-synaptic neurexin-neuroligin adhesion complex. This decreases the apposition of presynaptic RIM and postsynaptic AMPA receptors, as shown by dual-color *d*STORM, thus leading to impaired synaptic transmission (Haas et al., 2018). Other molecular adhesion complexes, such as those formed between Caspr2-Contactin-2, ephrin–ephrin receptors, and cadherins are also likely to play a role in trans-synaptic organization but remain to be studied in detail by SRM at central mammalian synapses.

3D-STORM and STED also revealed that RIM1, Munc13-1, ELKS, and RIM-BP2 are placed as close to the presynaptic membrane as Piccolo and Bassoon and essentially localized at the active zone of murine synapses, where they form a large protein complex beneath the membrane (Dani et al., 2010; Grauel et al., 2016; Tang et al., 2016; Wong et al., 2018). At hippocampal synapses, using multi-color time-gated STED (gSTED) with a lateral resolution of ∼50 nm, RIM-BP2 was found to be part of the active zone scaffold and to form a complex with the priming factors RIM and Munc13 (Grauel et al., 2016). Deletion of RIM-BP2 causes mild changes in the localization of Ca_v_2.1 calcium channels relative to Bassoon. This results in a moderate reduction in release efficiency but leads to pronounced alterations in short-term plasticity. Therefore, by contributing to the proper localization of Ca_v_2.1 at active zones, RIM-BP2 fine-tunes the calcium-secretion coupling, with important consequences for synaptic output. RIM was shown to bind to the membrane phospholipid phosphatidylinositol 4,5 biphosphate (PIP2) via its C2B domain in a calcium-independent manner (de Jong et al., 2018). The deletion of RIM significantly reduces Munc13 and primed vesicles at actives zones, as assessed by STED. A C2B deletion mutant still localizes to active zones and can revert both Munc13 levels and primed vesicles. However, it fails to rescue exocytosis, probably by mistargeting the PIP2-dependent release machinery away from PIP2 in the membrane (de Jong et al., 2018). The localization of RIM-BP2 clusters relative to Munc13-1 clusters displays synapse specificity in the hippocampus, with the average distance to the nearest cluster being over 50% larger at mossy fiber synapses than at CA3-CA1 synapses, as shown by multi-color gSTED with a lateral resolution of 50 nm (Hofmann et al., 2005). A greater distance between RIM1 and Ca_v_2.1 clusters was also observed in mossy fiber synapses, where RIM-BP2 deletion alters Munc13-1 cluster number and distribution, but not at CA3-CA1 synapses. These results reveal that, beyond the striking structural differences, distinct active zone nano-architectures may explain functional differences between the two synapse types. Yet, the determinants of these nano-architectural differences remain unexplained. In yet another study, 3D-STORM was used to show that Munc13-1 forms discrete supramolecular nano-assemblies at active zones of glutamatergic synapses in hippocampal neurons, whose number closely matches the number of release sites. These supramolecular complexes recruit syntaxin-1 and define the physical entities that constitute functional quantal release sites where vesicles can dock, prime, and fuse (Sakamoto et al., 2018). Their multiplicity at single active zones provides a purely presynaptic mechanism for setting synaptic weight across synapses.

Unlike the sub-millisecond neurotransmission operating at glutamatergic and GABAergic synapses, where specialized sites support a tight coupling between pre- and postsynaptic compartments, some neurotransmitters have a more widespread action through diffusion over large areas. Dopamine is an important neuromodulator that controls brain functions essential for reward, motivation, and the control of movement, and generally acts as a volume transmitter at much slower time scales than glutamate or GABA. However, fast and spatially localized dopamine signaling has also been observed (e.g., Howe and Dombeck, 2016), prompting the search for specialized dopamine secretion sites supporting fast signaling. Using 3D-SIM, several typical active zone scaffold proteins, including Bassoon, RIM, and ELKS, were identified in striatal dopamine axons. These proteins were also shown to be co-clustered in tyrosine hydroxylase (TH)-positive synaptosomes using multi-color STED, which also revealed that Bassoon colocalized with synaptobrevin-2-positive vesicles (Liu et al., 2018). However, the participation of RIM and ELKs in dopamine release were distinct from fast synapses, with RIM being essential and ELKS dispensable. This study also demonstrates that ∼30% of dopamine varicosities contain active zone-like release sites that could execute fast signaling, though most receptors seem to be localized outside synapses, meaning that dopamine would still typically act as a volume neuromodulator. Regardless, the existence of active zone-like dopamine release sites containing molecular players that are common to other synapse types could implicate dopaminergic dysfunction in diseases linked to mutations in release machinery components and typically associated with glutamatergic or GABAergic dysfunction.

### Synaptic Vesicle Ultrastructure and Dynamics

The fusion of synaptic vesicles with the plasma membrane to release neurotransmitters is the last step in a long chain of complex—and not yet fully understood—molecular events involving a large number of presynaptic players (Südhof, 2013). Vesicles fuse at the active zone, are endocytosed in a compensatory, coupled exo-endocytic process, and are subsequently refilled with neurotransmitter for reuse (Maritzen and Haucke, 2018). These processes imply vesicle movement within the presynaptic bouton, but their small size precludes imaging of single vesicles with conventional microscopy techniques. Therefore, the movement of vesicles toward the plasma membrane, of vesicle material at the membrane, and of the endocytosed vesicles back to the vesicle pool had not been investigated in detail prior to the advent of SRM. The first study to address these questions used STED microscopy at low-intensity excitation to achieve live imaging of fluorescently labeled synaptic vesicles inside the axons of cultured neurons, at speeds of 28 frames per second and a focal spot size of 62 nm (Westphal et al., 2008). Within presynaptic boutons, vesicles were mostly in a low mobility and constrained state with average speeds of ∼2 nm/ms, characterized by both diffusive and motor-driven non-directional movement; however, rapid movement along axons was also recorded. Vesicle “hot spots” were also observed, where vesicles remain temporarily trapped. Subsequent research, also using STED, showed that the relatively high level of vesicle mobility initially reported—which contradicted the accepted dogma of low vesicle mobility—was due to imaging of recently endocytosed vesicles, since resting vesicles imaged after a prolonged incubation were largely stationary (Kamin et al., 2010). Quite surprisingly, and contrary to hypothetical assumptions, vesicle mobility was not altered by electrical or high KCl stimulation (Westphal et al., 2008; Kamin et al., 2010), two manipulations that greatly accelerate vesicle fusion rates. The explanation for these behaviors could be rather simple; vesicles undergoing fusion are already docked to the membrane and part of an immobile pool, whereas moving vesicles have enough motility to reach active zones to replenish the releasable pool. Therefore, changes in vesicle mobility may not be a prerequisite to sustain synaptic transmission, but it should be noted that technical issues related with the time at which imaging was possible after stimulation may have hampered detecting very immediate changes in mobility (Kamin et al., 2010). After fusion, the vesicle material was also found to have a limited motion at the membrane, contradicting the notion of its free diffusion out of synapses. Inhibition of synaptic activity, however, results in decreased mobility of recently endocytosed vesicles (Kamin et al., 2010). These results also question the physiological significance of the resting vesicle pool, since their immobility precludes any participation in the release process, except maybe under non-physiological stimulation conditions. A bi-directional shuttling between the membrane and an inner vesicle pool was also observed at hippocampal synapses by single-molecule localization microscopy using a vesicular Glutamate transporter 1 (vGlut1)-pHluorin fusion protein, with a localization precision of ∼27 nm. The retention of vesicles at the plasma membrane was shown to depend on myosin V acting as a tether instead of a motor, that also plays a role in refilling the release sites during repetitive stimulation, and in regulating the spatial distribution of release at more central sites in the synapse (Maschi et al., 2018). These results pave the way toward understanding the mechanisms involved in making vesicles available for release and in refilling release sites.

The existence of multiple release sites per active zone has long been put forward based on indirect estimates from electrophysiology experiments and on electron microscopy data showing the presence of docked vesicles at multiple active zone locations. Indeed, multivesicular release has been demonstrated at many excitatory and inhibitory brain synapses (reviewed in Rudolph et al., 2015), and occasionally observed by electron microscopy at snap-frozen hippocampal synapses (Abenavoli et al., 2002). SRM techniques have enabled the direct visualization of vesicle fusion events at central mammalian synapses and estimation of the number of functional release sites at individual active zones. By combining PALM and single-molecule localization, it was shown that vesicle fusion sites were coincident with RIM nanoclusters (Tang et al., 2016). However, vesicle fusion sites were found widely distributed throughout the active zones (Maschi and Klyachko, 2017; Maschi et al., 2018) and to undergo repeated reuse, though there is an activity-dependent reduction in reuse and relocation to the active zone periphery (Maschi and Klyachko, 2017). This reduction in reuse may reflect rate-limiting steps such as the availability of docking/priming sites for new vesicles (Neher, 2010) while relocation of release sites could represent a mechanism for minimizing postsynaptic receptor saturation to maintain transmission fidelity. Additionally, action potential-evoked release is more restricted to central, RIM-rich areas of active zones, compared to spontaneous release (Tang et al., 2016; but see Kusick et al., 2018). This raises the hypothesis of different fusion mechanisms operating across the presynaptic active zone, which may become permissive with repeated use, for example, resulting from sustained calcium elevation. Therefore, it would be interesting to investigate if more peripheral spontaneous fusion events colocalize preferentially with scaffold clusters other than RIM. A more recent study using 3D-STORM also demonstrated the existence of multiple quantal release sites at excitatory synapses, that are defined by the presence of Munc13-1 nano-assemblies. Though variable between synapses, these were stable at individual synapses (Sakamoto et al., 2018). Collectively, these results have shown a variable number of active release sites, averaging around 10 per active zone, a number that agrees rather well with the number of docked vesicles found at hippocampal synapses and shown to be the morphological correlate of fusion-competent vesicles (Schikorski and Stevens, 2001). However, there seems to be an unexplained discrepancy between the restricted localization of scaffold nanoclusters at the center of the active zones and the more widespread distribution of release sites throughout the active zone. Explanations could lie in differences in thresholding for cluster detection, and labeling and detection methods across studies. It also remains to be determined if the sites of morphological vesicle docking and vesicle fusion are one and the same, and further refinements are needed to provide a clearer picture of the vesicle fusion process at active zones.

In order to maintain efficient, sustained, synaptic activity vesicles must recycle fast enough, and clearance of release sites for subsequent fusion is rate-limiting (Neher, 2010). Secretory carrier membrane proteins (SCAMPs) are a family of conserved membrane proteins involved in membrane trafficking events and found, among others, in secretory granules, transporter vesicles, and synaptic vesicles. SCAMP5 is highly enriched in synaptic vesicles and a candidate gene for autism (Castermans et al., 2010), though its synaptic function has remained elusive. In cultured neurons, dual-color STORM revealed that SCAMP5 plays an important role in endocytosis and release site clearance, since newly exocytosed synaptotagmin does not relocate to perisynaptic areas when SCAMP5 is knocked down (Park et al., 2018). This leads to slower recovery of releasable synaptic vesicles and to synaptic depression, which could underlie synaptic dysfunction in the context of at least some forms of autism.

The ultrastructure of synaptic vesicles themselves in brain synapses has also been resolved by SRM at a resolution comparable to that obtained by immunogold electron microscopy, but with vastly improved label density, using multi-color caged *d*STORM (a variation of *d*STORM that employs spectral demixing and reductive dye caging; Lampe et al., 2012). By superimposing many ring-like structures labeled for either VGlut1 or clathrin, it was possible to reconstruct rings of 41 and 56 nm, consistent with the sizes of synaptic vesicles and endocytic intermediates seen by transmission electron microscopy, respectively (Lehmann et al., 2015). The drawback of this approach is that individual vesicles at synapses cannot be detected in sufficient detail, as with electron microscopy. In addition to small synaptic vesicles used to release neurotransmitters, neurons also secrete neurotrophins and neuropeptides in a regulated manner from dense-core vesicles (DCVs) from both axons and dendrites. *d*STORM and STED were used to estimate the number of DCVs in cultured neurons and their axonal density *in vivo*, respectively (Persoon et al., 2018). DCVs were found to fuse in dendrites and, preferentially, in axons, but the nanoscopic organization of the release sites was not investigated. This would be very interesting, though, to see if the nanoscopic organization of such sites in neurons resembles the active zones where small synaptic vesicles fuse. Finally, using dual-color *d*STORM with a resolution of ∼20 nm, it was shown that the endogenous neurotrophin, brain-derived neurotrophic factor (BDNF) was contained in small granule-like clusters of ∼60 nm, mostly within the presynapse of glutamatergic—but not GABAergic—terminals in long-term cultured hippocampal neurons (Andreska et al., 2014). Retrograde BDNF signaling has been shown to exert important roles in the brain (e.g., Choo et al., 2017). This SRM study demonstrates that most BDNF is, in fact, available for anterograde release at the synaptic sites where it is known to exert a strong neuromodulatory effect.

### Vesicle Fusion Machinery and Calcium Channels

The tethering and docking of synaptic vesicles are followed by vesicle fusion, orchestrated by the SNARE complex together with auxiliary proteins such as Munc18 and complexins, and triggered by a calcium sensor of the synaptotagmin family (Jahn and Scheller, 2006). A large body of evidence on the nanoscopic organization of the exocytotic machinery has been obtained from neuroendocrine cells or at the Drosophila neuromuscular junction using SRM techniques. Surprisingly, though, given the large interest in understanding the nanoscale organization of the release machinery at central mammalian synapses, SRM studies in these structures are quite scarce. The distribution of SNAP-25, syntaxin-1, and Munc18 were resolved in cultured neurons using a dual-color stochastic method with a resolution of 13 nm, showing that they colocalize at axonal membranes in clusters of 100 nm or less (Pertsinidis et al., 2013), though it is unclear if these correspond to active zones. However, STED showed that SNAP-25 and syntaxin are, as expected from their functions, enriched at synapses (Wilhelm et al., 2014). Ablation of syntaxin expression causes complete loss of the Munc18-1/SNAP-25 association and loss of Munc18-1 into the cytoplasm. This shows that Munc18-1 associates with SNAP-25 through syntaxin-1 (Pertsinidis et al., 2013), the only t-SNARE to possess a transmembrane domain. In cortical neurons, *d*STORM and PALM revealed the localization and dynamics of syntaxin-1a and Munc18-1 at synapses, as identified by co-labeling for synapsin (Kavanagh et al., 2014). Munc18-1 is mobile along axons, displaying directed movement and traveling long distances between synapses, while exhibiting a restricted movement in puncta. Consistent with its binding to syntaxin, the speed of Munc18-1 increases upon disruption of its interaction with syntaxin-1a, as shown by single-particle tracking PALM. Also in cultured neurons, multi-color gSTED showed that the distance between the synaptic vesicle-anchored, SNARE complex protein synaptobrevin 2, and the scaffold protein intersectin 1, present at active zones, is reduced during synaptic activity, indicating that the latter directly associates with the SNARE complex during exocytosis (Jäpel et al., 2020). This association is key for the clearance of release sites, thereby providing a mechanism for exo-endocytic coupling that allows synapses to sustain high-frequency neurotransmission. One potential issue in detecting the proper localization and interactions of SNARE proteins (or others) at the nanoscale is not only the large size of the antibodies used for labeling but also their potential to form aggregates, which can cause localization/distribution errors in SRM. Using the much smaller camelid single domain antibodies (or nanobodies) combined with dual-color STED, SNAP-25 and syntaxin-1a were shown to cluster at synapses of cultured neurons, with syntaxin-1a presenting more homogeneous cluster sizes. Considerable extrasynaptic localization was also detected, implying that, while essential for vesicle fusion, these proteins are not likely to play major roles in defining the sites of exocytosis (Maidorn et al., 2019). However, their recruitment to synapses upon stimulation suggests an active functional role, and it would be interesting to investigate whether a substantial extrasynaptic localization of SNARE proteins is also observed in intact brain tissue.

Calcium channels are crucial players in neurotransmitter release, since they provide the trigger for the exocytotic machinery to execute vesicle fusion. Their localization in respect to both fusion sites and the release machinery is considered essential for a tight coupling between action potential-driven calcium influx and neurotransmitter release (Eggermann et al., 2012), which, in turn, is required for high-fidelity synaptic transmission. However, a loose coupling has been reported at hippocampal synapses (Vyleta and Jonas, 2014) and, indeed, SRM has shown that calcium channel distribution can be quite variable at mammalian synapses. At cerebellar parallel fiber synapses, dual-color *d*STORM with a localization precision of ∼13 nm showed an enrichment of Ca_v_2.1 channels at active zones, close to Bassoon and metabotropic glutamate 4 receptors (mGluR4), but also outside the active zones (Siddig et al., 2020). The proximity of Ca_v_2.1 to mGluR4 is also closer than expected for a random distribution, suggesting a functional interaction (see discussion below). At excitatory hippocampal synapses, multi-color gSTED showed that Ca_v_2.1 clusters significantly segregate from Bassoon clusters (Grauel et al., 2016). Similar observations were made using *d*STORM, that additionally showed no overlap of Ca_v_2.1 with RIM clusters (Glebov et al., 2017), with spatial segregations as large as 50 nm. These results are surprising since RIM was shown to tether calcium channels through a direct interaction with their PDZ domain (Kaeser et al., 2011), which is likely incompatible with the range of segregation distances observed. Again, labeling densities and detection thresholds could account for smaller measured protein cluster sizes, or to failure in detecting calcium channels in close proximity to RIM clusters, if they are too few, leading to apparent spatial segregation. However, indirect interactions of RIM with calcium channels, mediated by RIM-BPs (Hibino et al., 2002; Grauel et al., 2016), could also help explain this spatial segregation, if an intermediary link is present that would increase the distance between the two proteins. Interesting insight into how these proteins can organize at active zones came from the demonstration that RIM and RIM-BP can autonomously assemble into condensed complexes by liquid-liquid phase separation and cluster calcium channels into microdomains (Wu et al., 2019). It would be most interesting to demonstrate if additional active zone components also spontaneously tether around these assemblies to form active zone-like structures. One outstanding question has been whether calcium channels—or their activity—promote synapse assembly or, conversely, whether active zone proteins organize these channels at release sites. Using 3D-STORM, the nanoscale organization of RIM clusters relative to PSD-95 was shown to be unchanged in the absence of all three Ca_v_2 calcium channel subunits in cultured hippocampal neurons. Furthermore, STED showed that the presence and localization of the active zone proteins RIM, RIM-BP2, Liprin-α3, ELKS2, Bassoon, and Munc13-1 are unchanged by the absence of calcium channels, though some are even mildly upregulated (Held et al., 2020). Therefore, neither the organization of presynaptic active zone scaffold nano-domains, nor their trans-synaptic alignment with postsynaptic nano-domains, require the presence of calcium channels. Notwithstanding, the nano clustered organization of presynaptic calcium channels remains consistent with the concept of calcium microdomains, shaped by the distance of calcium channels to vesicle docking sites together with the diffusion and buffering of calcium (Neher, 1998), though how the calcium channel nanodomains and release sites are coupled still remains unclear. Rather surprisingly, calcium channels also present considerable mobility at the presynaptic membrane of hippocampal synapses (Schneider et al., 2015). Indeed, in cultured hippocampal neurons, single particle tracking PALM with a localization accuracy of ∼27 nm revealed that a large proportion (∼60%) of exogenously expressed Ca_v_2.1 channels are mobile in the presynaptic membrane, though their movement is confined. Calcium channel movement was shown to be reduced by buffering basal calcium but unchanged by its rise during synaptic activity. Importantly, STED showed that RIM and Bassoon clusters scale with Ca_v_ channel number in a way that allows active zones to maintain channel density and mobility (Schneider et al., 2015). These mechanisms may allow the cooperation between calcium domains and equalize the probability of release among docked vesicles. It would be interesting to see if similar observations are made at other types of synapses and, quite importantly, at synapses in intact tissue.

### Presynaptic Neurotransmitter Receptors

Several classes of neurotransmitter receptors, including glutamate, GABA, and cannabinoid receptors, have been known for many decades to have a prominent presynaptic localization where they play important regulatory functions as auto- or heteroreceptors (e.g., Draguhn et al., 2007; Pinheiro and Mulle, 2008; Banerjee et al., 2016). However, detailed information on their specific subunits/assemblies, density, trafficking, and precise localization at presynaptic sites is scarce, and their very existence is, in some cases, still debated. One of the earliest SRM studies in brain tissue identified the presence of GABA_B_R1 receptors at active zones of glutamatergic synapses by STORM, with an axial localization overlapping that of the presynaptic membrane (Dani et al., 2010). Retrograde endocannabinoid signaling through presynaptic CB1Rs is a widespread mechanism of modulation of synaptic transmission and plasticity (Ohno-Shosaku and Kano, 2014) that displays marked synapse-specific differences (Miles et al., 1996). Using multi-color 3D-STORM with a lateral localization precision of 6 nm and 41 nm axially, presynaptic CB1Rs were found to have a uniform distribution on GABAergic terminals in acute hippocampal slices, though they were more abundant on perisomatic than on dendritic interneuron terminals (Dudok et al., 2015). A higher CB1/Bassoon ratio was observed at perisomatic synapses, which may allow the more efficient coupling to the modulation of the release machinery, thereby explaining their higher sensitivity to endocannabinoid signaling. Chronic treatment with Δ^9^-tetrahydrocannabinol (THC) causes internalization and loss of CB1 receptors at these terminals, as assessed by 3D-STORM (Dudok et al., 2015), thereby explaining the reduced efficacy of cannabinoids on GABA release following THC administration (Hoffman et al., 2007). Quite interestingly, at these same CB1-positive terminals in the hippocampus, dual-color 3D-*d*STORM identified the presence of ribosomes within 25–400 nm of the presynaptic membrane (Younts et al., 2016). Here, they integrate CB1R signaling to mediate the protein synthesis-dependent long-term depression (LTD) of GABAergic transmission through cap-dependent local presynaptic translation (Younts et al., 2016). The presence of ribosomes in the presynaptic compartment was also identified in most glutamatergic and GABAergic synapses of both cultured hippocampal neurons and brain slices using expansion microscopy (Hafner et al., 2019), indicating that local protein synthesis is ubiquitously present at synapses. Another type of neurotransmitter receptor frequently found at presynaptic sites are G_i/o_-coupled metabotropic glutamate receptors (mGluRs) that exert a critical inhibitory function as auto- or heteroreceptors (Huang and Thathiah, 2015). Using dual-color *d*STORM with a localization precision of 13 nm, a recent study obtained a detailed characterization of presynaptic mGuR4R number, stoichiometry, and spatial arrangement at parallel fiber synapses in the cerebellum (Siddig et al., 2020). At these synapses, mGluR4 was found concentrated within the active zones, which contained an average of 35 mGluR4 subunits mostly arranged in small nanoclusters of 1–2 subunits (average, 25 nanoclusters of 1.4 subunits), though high variability was observed. mGluR4 nanodomains were found close to Munc18-1 (30 nm) and Ca_v_2.1 (65 nm), suggesting that these proteins might co-exist in functional macromolecular complexes that influence neurotransmission by direct regulation of the exocytotic machinery and calcium channel function. While scarce, given the wealth of reports on their existence and functions, overall, these studies highlight the diversity of localization and nanoscopic organization of presynaptic neurotransmitter receptors relative to the active zones, which will have important consequences for presynaptic modulation. Further studies are needed to understand where other presynaptic neurotransmitter receptor types localize to function in the modulation of neurotransmission.

### Other Presynaptic Elements

Besides the obvious interest in studying the nanoscale localization, abundance, and dynamics of active zone proteins, various other presynaptic elements have been researched using SRM imaging at mammalian presynapses. The first application of STED to investigate synaptic organization achieved a lateral resolution of 40 nm at the calyx of Held synapse, a giant glutamatergic terminal located in the auditory brainstem that contains hundreds of individual active zones. Here, VGlut1, synaptophysin, Rab3A, and synapsin signals were shown to be consistent with a vesicular distribution, although synapsin was absent from a subpopulation of vGlut1-positve vesicles (Kempf et al., 2013). Using N-SIM, the presence of c-Jun NH2-terminal protein kinase (JNK)—mainly recognized as being postsynaptic—was found colocalized with synaptophysin in mouse purified cortical synaptosomes, where it was coupled to the activity of presynaptic NMDA receptors (Biggi et al., 2017). Presynaptic NMDARs, once considered an exception, are now believed to be quite widespread in the brain and to play important roles in modulating synaptic transmission and plasticity (Bouvier et al., 2015). However, anatomical data for their localization comes mainly from immunogold EM, which fails to report accurate receptor densities and colocalization with other synaptic components. It is, therefore, unfortunate that the presence and precise localization of the NMDARs in question were not investigated by SRM in the study by Biggi et al. (2017), which could also lend support to their functional presynaptic interaction with JNK. Using a combination of multi-color STORM and multi-color STED, gamma secretase, the enzyme responsible for the last processing step of the amyloid precursor protein, was found to localize in close proximity (down to <10 nm) of presynaptic synaptophysin-positive vesicles in hippocampal neurons (Schedin-Weiss et al., 2016), but to be absent from docked synaptic vesicles. This suggests that gamma secretase localizes to intracellular membranes/vesicular structures other than synaptic vesicles. Its presence is also very variable, with some synapses containing almost no labeling. Finally, despite being predominantly nuclear, the small ubiquitin-like modifier (SUMO) 2/3 protein was found to colocalize with the presynaptic protein synaptophysin using N-SIM (Colnaghi et al., 2019), although no attempt was made to further resolve its nanoscopic organization relative to active zones. The functions of RIM1α, synaptotagmin1, syntaxin1A, synapsyn1a, and possibly other proteins are modulated by SUMOylation (Henley et al., 2018), and demonstrating the presence of SUMO proteins at presynapses was a missing piece of the puzzle, though it requires further investigation.

### Outlook

Almost 500 proteins, from a wide variety of functional categories, were identified in biochemically purified presynaptic fractions of central synapses (Boyken et al., 2013; Weingarten et al., 2014); about half of these are from the active zone. However, only a small amount has ever been studied in detail by SRM, and the vast amount of information that can still be gathered using these techniques will be crucial for a better understanding of presynaptic function. For example, different synaptotagmin isoforms contribute to the full capacity of release at central synapses (e.g., Bacaj et al., 2013, 2015), but it remains debated if they are co-localized in vesicles, sorted to distinct vesicle populations, or even whether some may act from the plasma membrane side. Another C2 domain protein akin to synaptotagmins is Doc2b, whose precise role at central synapses is still controversial. Doc2b has been postulated as a high-affinity calcium sensor for spontaneous neurotransmitter release (Groffen et al., 2010) and traffics to the plasma membrane in a calcium-dependent manner in chromaffin cells (Groffen et al., 2004, 2006), where it plays important roles in DCV priming (Pinheiro et al., 2013; Houy et al., 2017). However, its precise localization at mammalian presynapses, and whether it displays calcium-dependent membrane translocation in this nano-environment—important to understand its synaptic function—have not been determined. Additionally, despite the plethora of functional and biochemical evidence for the existence of presynaptic GABA, NMDA, kainate, and, to a lesser extent, AMPA receptors, their study at presynaptic structures using SRM has attracted surprisingly little interest. However, this would be highly relevant to complement existing functional studies, since their localization relative to active zone components, molecular composition, surface trafficking, and whether they are concentrated in highly organized nanodomains—like their postsynaptic counterparts—are likely to influence how they modulate presynaptic activity. The results obtained from studying vesicle fusion by SRM also raised interesting questions regarding the local segregation of release sites and the tethering of the active zone scaffold proteins to the membrane, since none possesses a transmembrane domain. One key element could be the membrane phospholipid PIP2. PIP2 is required for the function of many components of the vesicle fusion machinery including syntaxin, Munc13, calcium channels, and synaptotagmin (Bai et al., 2004; Chun et al., 2010; Suh et al., 2010; Van Den Bogaart et al., 2011). RIM1, whose nanodomains at the active zone define vesicle release sites, binds to PIP2 via its C2B domain (de Jong et al., 2018), thereby targeting the release machinery to sites where this lipid is present and necessary for fusion efficiency. Visualizing the nanoscale co-distribution of PIP2 and RIM (or RIM-ΔC2B) at active zones and acutely manipulating PIP2 levels (for example, using the recently developed caged PIP2; Walter et al., 2017) could help to clarify if this phospholipid is the orchestrator of active release sites at the membrane. Several other scaffold proteins, including Bassoon and Munc13, also contain C2 or other lipid-binding domains; whether their interaction with PIP2 also contributes to active zone organization remains to be determined. These, and many other outstanding questions, could probably find an answer by imaging in the nanoscale domain using SRM techniques.

## Perspectives for SRM of the Presynaptic Compartment

Despite the large accomplishments of “classical” SRM techniques, each has its weaknesses or limitations, and continued research into ways of further improving their resolving power, speed, or imaged area has led, in recent years, to the development of both entirely new concepts and variations of existing ones. Combining different SRM methods, or SRM with other imaging or experimental approaches, has proven effective at harnessing the advantages of each. For example, STED microscopy has been combined with expansion microscopy (ExSTED; Gao et al., 2018; Kim et al., 2019), allowing further resolution gains to under 10 nm. This approach could be particularly relevant in the extremely crowded space of synaptic compartments, particularly if using probes that are smaller than antibodies. By enabling significant molecular decrowding and fluorophore separation due to sample volume expansions of up to 1000 fold (Truckenbrodt et al., 2018), the recently developed X10 expansion microscopy alone can produce super resolution images on standard epifluorescence microscopes that rival those obtained in commercial implementations of STED or STORM (Figure 2). If combined with these physics-based SRM techniques, X10 microscopy may allow resolution gains down to the size of single fluorophores and the generation of extremely accurate maps of protein distribution and density. Expansion microscopy is also enormously advantageous since it’s cheap to implement and allows significant resolution gains without the need for specialized equipment, technical knowledge, or complex analysis software, making it accessible to virtually any lab with an epifluorescence microscope. It is also compatible with thick samples and standard fluorophores, but cannot be used for live imaging. Also noteworthy is the combined use of PALM and uPAINT with 3D-STED or SUSHI imaging methods onto a single microscope platform (Inavalli et al., 2019). By combining the strengths of deterministic and stochastic SRM methods, this system allows the simultaneous investigation of both the nanoscale morphology of synapses and the localization and dynamics of synaptic proteins in living samples and opens the possibility of applying a similar approach using other SRM techniques. Finally, approaches using correlative SRM and electron microscopy have succeeded in combining the superior resolution of the electron microscope with the molecular specificity and ability to provide quantitative data on the number, distribution, and size of protein complexes afforded by SRM techniques (Nanguneri et al., 2012; Kim et al., 2015; Johnson and Kaufmann, 2017; Ando et al., 2018; Dietz and Heilemann, 2019; Franke et al., 2019). However, SRM or other imaging techniques cannot decipher the complexity of synapses and neuronal and brain function on their own, since images alone will not tell the whole story. The combination of SRM with electrophysiology (Chéreau et al., 2017; Yadav and Lu, 2018; Schmidl et al., 2019), digital holography (Lauterbach et al., 2016), and optogenetics (Dani et al., 2010; Glebov et al., 2017) holds great promise toward correlating functional and structural/molecular aspects of synapse function.

**FIGURE 2:** X10 expansion microscopy can achieve super resolved images on a conventional microscope. **(A)** Immunostaining for the peroxisome membrane protein Pmp70 in neurons, imaged before expansion by confocal, STED, or STORM microscopy, and by standard epifluorescence microscopy after classical 4x sample expansion or X10 sample expansion. The last panel shows the X10 image after deconvolution. Scale bar, 100 nm. **(B)** Representative immunostaining images for postsynaptic PSD95 (magenta) and presynaptic RIM1/2 (green) proteins in cultured neurons at an expansion factor of 10.4x. Nanocolumns of aligned pre- and postsynaptic proteins are indicated by arrowheads. Scale bars: 500 nm (upper panel) and 200 nm (lower panels). Adapted, with permission from Truckenbrodt et al. (2018).

Although some SRM techniques have reached a high level of maturity and are now offered as commercial solutions, emerging new concepts are again pushing the boundaries of resolution and/or speed. MINFLUX nanoscopy, for example, can probe single-molecule emitters with a donut-shaped illumination pattern and resolve molecules distanced by as little as 6 nm with a precision of 1 nm, while requiring a much lower photon budget than common centroid-based methods (Balzarotti et al., 2017) (Figure 3). However, unlike STED, where the donut-shaped illumination pattern is used both to generate the fluorophore state transitions and for their localization, in MINFLUX it is used only for localization. The concept is compatible with 3D multi-color labeling applications (Gwosch et al., 2020), has been extended to the use of sinusoidal illumination patterns (Reymond et al., 2019; Cnossen et al., 2020), and could replace the now common SRM methods, eventually allowing molecular resolution in lensless designs (Balzarotti et al., 2017). Applied to neurons and synapses, these methods could push our understanding of their intricate nano-organization and dynamics down to molecular resolution while limiting phototoxicity concerns, particularly if they can be made compatible with *in vivo* deep-tissue imaging.

**FIGURE 3:** MINFLUX nanoscopy of labeled DNA origamis allows resolving molecules only 6 nm apart. **(A)** Arrangement of up to nine on-off switchable Alexa Fluor 647 fluorophores on the DNA origami with an 11 nm spacing (in gray are depicted those that remained in the off state throughout the measurement). **(B)** Spatial binning (bin size, 0.75 nm) of direct MINFLUX localizations renders a nanoscopic image of the origami from events yielding > 500 photons. **(C)** Simulated ideal PALM/STORM image of the origami using detections of 500 photons. **(D–F)** Similar representations as in **(A–C)** but for the smaller DNA origami depicted in **(D)**. Events with under 100 detected photos were discarded. Adapted, with permission from Balzarotti et al. (2017).

## Conclusion

By harnessing the resolving power of super-resolution optical microscopy, our understanding of synapse structure and function has taken big leaps in recent years. With the incessant quest for further refinements in terms of better hardware, increasingly powerful processing algorithms (e.g., Xu et al., 2017), or deep learning strategies (Ouyang et al., 2018; Wang et al., 2019; Jin et al., 2020), fluorophores with improved or tailored photophysical properties (e.g., Minoshima and Kikuchi, 2017; Thiel and Rivera-Fuentes, 2018; Halabi et al., 2019; Kozma and Kele, 2019; Velde et al., 2019; Xu et al., 2020), and, quite likely, yet new and revolutionary technical approaches altogether, the limits of what can be resolved today are bound to keep shrinking. In parallel, the evolution of strategies for high-throughput SRM are allowing faster imaging of increasing numbers of simultaneous targets over larger sample areas (Guo et al., 2019; Mahecic et al., 2019). We look forward to seeing—in super-resolution—what synapses and other neuronal structures will resemble in the future.

## Author Contributions

All authors listed have made a substantial, direct and intellectual contribution to the work, and approved it for publication.

## Conflict of Interest

The authors declare that the research was conducted in the absence of any commercial or financial relationships that could be construed as a potential conflict of interest.
